# An Intelligent System for Detecting Abnormal Behavior in Students Based on the Human Skeleton and Deep Learning

**DOI:** 10.1155/2022/3819409

**Published:** 2022-06-27

**Authors:** Yourong Ding, Ke Bao, Jianzhong Zhang

**Affiliations:** Wuxi Institute of Technology, Wuxi, Jiangsu 214121, China

## Abstract

With the use of an intelligent video system, this research provides a method for detecting abnormal behavior based on the human skeleton and deep learning. To begin with, the spatiotemporal features of human bones are extracted through iterative training using the OpenPose deep learning network and the redundant information of human bone facial features is reduced in the feature extraction process, effectively reducing the time it takes to identify and analyze abnormal behavior. The collected human skeleton features are then classified using a graph convolution neural network to reduce the computational complexity of the behavior identification algorithm, and the sliding window voting method is used to further improve the accuracy of the behavior classification in practical application, resulting in the diagnosis and classification of abnormal behavior of students under video surveillance. Finally, using the self-built student trajectory data set and the INRIA data set, simulation analysis is performed, and the practicality and superiority of the proposed method for abnormal behavior detection is confirmed by comparing it to the existing abnormal behavior recognition methods. The proposed method for detecting anomalous behavior in a self-built database and INRIA data set has a high accuracy of more than 99.50 percent and a high processing efficiency rate.

## 1. Introduction

The society is developing rapidly, and the population is large and increasingly dense. Traffic accidents, fights, and other socially unstable incidents occur from time to time, and even terrorist attacks occur. Social security needs to be greatly enhanced. The number and coverage of surveillance cameras in transportation systems and public places are also increasing year by year, and cameras are basically found in every aspect of people's daily lives. In order to ensure people's safety, the camera can simulate human eyes so that they have the ability to “see.” Computers simulate human brains with decision-making abilities. The computer obtains the video data through the surveillance camera for calculation and analysis, so as to understand the picture content in the surveillance scene, so as to realize the detection, identification, early warning, and alarm of abnormal behavior. As a kind of transportation equipment, escalators are widely used in shopping malls, office buildings, schools, and other public places to facilitate the people's travel. Especially for students, as a specific group of the society, because of their own sense of autonomy and physical condition is still immature, a variety of hand lift safety accidents are prone to occur. At the same time of enhancing students' safety awareness, it is more necessary to monitor the escalator to stop the occurrence of safety accidents in time; in addition, by monitoring whether there are students on the escalator, it can also avoid no idling of the escalator, so as to save energy and prolong the life of the escalator, and realize fine management by counting the passenger flow of the escalator [1].

Intelligent video monitoring system (IVMS) has the characteristics of low cost, accuracy, and stability, and has been paid more and more attention in the field of public security [2, 3]. Passenger abnormal behavior recognition is an important application in IVMs, which can detect and track moving targets through video sequences to analyze the target behavior [4–6], detect abnormal behavior fragments, and then identify abnormal behavior categories. When students take the escalator, abnormal behaviors such as falling, climbing the handrail, probe, and hand probing can cause serious safety accidents. Therefore, it is of great significance to apply IVMs to accurately and stably identify various abnormal behaviors [7, 8].

Traditional abnormal behavior recognition methods such as hidden Markov models can only recognize specific actions in a single, simple environment, and are easily affected by environmental interference in a complex environment, which will reduce the recognition rate. Based on image acquisition technology and artificial intelligence technology, the collected images are input into a multi-layer network model composed of convolution for training, feature extraction of image signal data, and continuous learning based on their own network to improve student shape recognition performance and effectively guarantee the safety of students [9, 10].

## 2. Related Works

Due to a lack of safety awareness, students as a distinct group of society cause escalator accidents. Many researchers have conducted study on deviant behavior analysis when riding escalators as the precision of intelligent monitoring systems has improved and the maturity of image analysis algorithms has grown.

Traditional aberrant behavior recognition is constrained by ambient elements like light and shadow, and has issues like imprecise recognition and low processing efficiency [11]. The direction change of human ellipse fitting can be used to identify abnormal behavior in literature [12], but it can only be used in a simple environment; in literature [13], a Gaussian mixture model and filtering method are used to detect moving targets, extract fusion features, analyze target posture, and accurately recognize indoor falls and paralysis behaviors in real time. However, precisely modeling the background in complicated scenarios is difficult, lowering the identification rate. The use of recursive filtering to get target characteristics in literature [14] can solve the problem of difficult modeling of complex backgrounds, but the amount of computation is considerable and cannot match real-time requirements. Aberrant behaviors can be detected in real-time using the Hidden Markov model; however, the sorts of abnormal behaviors cannot be identified [15]. The human body is identified by filtering channel features and features are retrieved by Hough direction calculator to identify a variety of abnormal behaviors, according to the literature [16], but the abnormal behavior sequence must be segmented in preparation.

To recognize abnormal behavior, spatial and temporal features that can represent human motion can be retrieved from the original image data using deep learning theory [17–19]. The spatiotemporal point of interest feature [20], silhouette feature [21], optical flow feature [22], depth feature [23], and human two-dimensional skeleton feature are some of the most widely used features. Kinect [24], a prominent abnormal behavior analysis technology at the moment, can easily extract the two-dimensional skeleton of the human body. Through iterative training and learning, a deep convolution neural network can efficiently extract feature information from the processing data set [25, 26] and realize behavior recognition and analysis. A dual residual convolutional network-based fall recognition algorithm was proposed in the literature [27]. The shallow and deep visual characteristics are fully integrated by nesting the residual network in the residual network, which reduces the impact of gradient disappearance during model training and improves the model's performance. Literature [28] calculates the optical flow field of sparse feature points using the Lucas–Kanade method, performs temporal and spatial filtering on the optical flow field, and detects anomalous behavior for the moving population using the graph convolutional neural network mode. A deep learning-based technique has been proposed in the literature [29]. The feasibility test was conducted using the VGG-16 model, which was trained on the open benchmark population data set. Through a cascaded network topology, literature [30] converts pretrained supervised FCN to unsupervised FCN based on convolution neural networks, which decreases the computational cost and enhances the real-time and accuracy of aberrant behavior detection.

The implementation of an intelligent video detection system and the use of intelligent approaches are critical for detecting inappropriate behavior in pupils when using escalators. However, contextual circumstances limit classic abnormal behavior, which has issues with identification accuracy and processing speed. This paper presents a method for detecting anomalous behavior in students based on the human skeleton and deep learning, based on previous anomaly detection research. The following are the major contributions:

1. The spatiotemporal properties of the human skeleton are retrieved using an OpenPose deep learning network to improve the accuracy and real-time of behavior recognition in escalator operation. The redundant information of face characteristics is eliminated during feature extraction, and the input original image is processed through the network to achieve end-to-end skeleton extraction results and effectively shorten the identification time.
2. This paper proposes a method based on graph convolution neural network to classify the collected human skeleton features, and uses sliding window voting method to further improve the classification accuracy in actual application, and finally realizes the video sequence diaphragm.

The remainder of this article is structured in the following manner. The second section introduces the abnormal behavior detection method's network model; the third section introduces the specific theoretical content and method implementation of the abnormal behavior detection method based on human skeleton and deep learning; the fourth section introduces the feasibility and optimality experimental simulation analysis of the proposed method using self-built and INRIA data sets; and the fifth section is the paper's conclusion.

## 3. The Proposed Model

Convolutional neural networks have difficulty extracting video features from huge numbers of frames and long-time sequences, but long-term and short-term memory networks have difficulty processing time sequence data in parallel and are slower. As a result, this article provides a skeletal action recognition model based on spatiotemporal relationship in order to better handle long-time video and meet real-time performance requirements, along with the characteristics of the two networks. The network may be used to recognize skeleton actions in long-term video and to recognize multi-person scenario behavior. The proposed method's flowchart is shown in Figure 1.

The abnormal behavior detection algorithm's ultimate purpose is to binary classify video sequences. First, the OpenPose pose estimation algorithm [31] extracts the 2D skeleton coordinates of the human body, and then the depth information of joint points is obtained using a monocular camera-based depth estimation method; then, the depth information and two-dimensional skeleton coordinates are combined to form three-dimensional skeleton data, and behavior recognition is performed using the skeleton data; finally, the skeleton recognition model is proposed based on the spatiotemporal relationship method.

## 4. Method and Implementation

### 4.1. Video Image Capture

The installation position of the escalator surveillance camera in a school is shown in Figure 2. Use a 3.6 mm focal length camera to shoot from diagonally above the escalator to ensure a clearer image.

The real video data are all scenes of passengers taking the escalator normally. There are many videos, and some video frames are intercepted for transfer learning of pedestrian detection models. The abnormal behavior was simulated by student volunteers on escalators in different scenes (air-floor, semi-outdoor). Affected by the camera's shooting angle and viewing angle, the maximum number of passengers in the escalator monitoring image is 5. The algorithm in this paper is not applicable to extreme situations with severe occlusion. For example, in the case of too many people, the passengers behind are blocked by a large area. And in a two-person scene, the person in front is relatively large, completely obscuring the person behind, etc. These situations will lead to missed detection of blocked passengers or most of the key point extraction results are missing (people who are not blocked in front have little influence). Therefore, in the volunteer simulation, this article only considers sparse scenes and crowded scenes where the occlusion is not serious. The videos simulated by the experimental volunteers in this article include 7 types of behaviors in different environments: standing normally, falling forward, falling backward, climbing the handrail, extending the head to the escalator, extending the hand to the escalator, and leaning against the handrail. Environmental variables are light intensity and passenger density.

The movie is initially divided into 1613 segments for the anomalous behavior data set. Each segment lasts 20–30 seconds and covers the entire process of passenger behavior in various contexts. The short video is then separated into a training set and a validation set based on behavior and environmental characteristics in a 3 : 1 ratio. The training set and verification set of the graph convolutional neural network are then recovered from the key behavior frames. In this approach, the operation of dividing the video data set first and then capturing the picture is compared to capturing the image first and then dividing the image data set, which can prevent using the same short video for both the training and verification sets. It also guarantees that the training model does not overfit the validation data.

### 4.2. OpenPose Deep Learning Network

According to the method of skeleton extraction, the skeleton extraction network can be divided into top-down and bottom-up extraction. A human body detector must be used to determine the position of the human body in order to extract the skeleton from top to bottom. The skeleton is then extracted by detecting key points of the human body in each human body area. This method relies on the human body detector's performance, and the speed of skeleton extraction slows dramatically as the number of people in the image grows. The bottom-up skeleton extraction does not require the detection of the human body, instead detecting all of the key points in the image directly. Then, using the same person's key points, create a human body skeleton. This method's skeleton extraction speed is unaffected by the number of people present, and the skeleton can be extracted quickly even when there are many. However, determining the relationship between the key points and the human body to which they belong is difficult. OpenPose presents Part Affinity Fields (PAFs) to communicate the relevant information between key points of the human body and the human body to which it belongs as a solution to this challenge. Each pixel corresponds to a two-dimensional vector in the PAFs, which are the same size as the original image. By connecting two adjacent key points in a straight line, you can encode the position and direction of the torso. The likelihood that the two key points can be joined to generate a human body torso is then calculated by adding the inner product of the PAFs vector and the connecting vector of all pixels on the segment connected by any two key points. The foundation for subsequent abnormal behavior detection and recognition is accurate, real-time, and stable skeleton extraction. Deep learning methods extract human skeletons more accurately and consistently than traditional image processing or machine learning methods. It creates a skeleton extraction network by iterative training, processes the input original images through the network, and outputs the skeleton extraction results from start to finish. Skeleton extraction networks have been regularly enhanced and put forward one after another as deep learning technologies have progressed. The OpenPose deep learning network used in this paper is one of them. It is a deep learning network that considers real-time performance and can accurately and consistently extract the human skeleton. It is the standard skeleton extraction network at this time, and it is widely used in the engineering area.

The network structure of OpenPose is shown in Figure 3. First, the first 10 layers of the VGG network are used as a pretrained convolutional neural network to generate a feature map set *F*. Then, input it into two branch networks, each branch network contains *T* stages. Each stage *t* of the first branch outputs a set of key point confidence maps *S*^*t*^. Each key point confidence map is a heat map corresponding to the key points of the human body, which is the same size as the original image. Each pixel value represents the confidence that the point belongs to the corresponding key point. Each stage *t* of the second branch outputs a set of PAFs map *L*^*t*^, corresponding to each segment of the human torso connected by key points. The input of the first stage is *F* and the output is *S*^1^ and *L*^1^. Starting from the second stage, the input of each stage *t* is the fusion feature map of *F* and the previous stage *S*^*t*−1^ and *L*^*t*−1^, and the output of *S*^*t*^ and *L*^*t*^.

At each stage, calculate the *L*_2_ norm of *S*^*t*^, *L*^*t*^ and *S*^*∗*^, *L*^*∗*^ as the loss function. Here, *S*^*∗*^ and *L*^*∗*^ are the real key point confidence map and real PAFs. Using the real label data, calculate according to

(1) $$\begin{array}{c} S_{j,k}^{*}\left(p\right)=\exp\left(\frac{-{\left|p-x_{j,k}\right|}_{2}^{2}}{\sigma }\right), \end{array}$$

(2) $$\begin{array}{c} S_{j}^{*}\left(p\right)=\underset{k}{\max}S_{j,k}^{*}\left(p\right), \end{array}$$

(3) $$\begin{array}{c} v=\frac{\left(x_{j_{2}k}-x_{j_{1}k}\right)}{{\left|x_{j_{2}k}-x_{j_{1}k}\right|}_{2}}, \end{array}$$

(4) $$\begin{array}{c} L_{c,k}^{*}\left(p\right)=\left\{\begin{array}{c} v,\text{0}\leq v\cdot \left(p-x_{j_{1}k}\right),\leq l_{c,k}\cup \left|v_{⊥}\cdot \left(p-x_{j_{1}k}\right)\right|\leq \sigma_{c,k},\\ 0,\text{otherwise,} \end{array}\right. \end{array}$$

(5) $$\begin{array}{c} L_{c}^{*}\left(p\right)=\sum_{k}L_{c,k}^{*}\left(\left(p\right)/n_{c}\left(p\right)\right), \end{array}$$

where *x*_*j*,*k*_ and *S*_*j*,*k*_^*∗*^(*p*) are the real position of the *j* key point of the *k* th person and the real confidence of the pixel point *p*, respectively. *σ* controls the smoothness of the distribution. *L*_*c*,*k*_^*∗*^(*p*), *l*_*c*,*k*_, and *σ*_*c*,*k*_ are the PAFs vector, torso length, and width of the torso of the *k* th person's section *c*, respectively. *v* and *v*_⊥_ are the torso unit vector and the vertical unit vector, respectively. *n*_*c*_(*p*) is the number of people with non-zero *L*_*c*,*k*_^*∗*^(*p*). Accumulate all stages to obtain the total loss function. Continuously optimize the total loss function through iterative training until the model converges to obtain the final network model. The network output is the *J* key point confidence level and the *C* segment trunk PAFs graph. The key points can be used as nodes in the bipartite graph, and the possibility *E* of connecting the two key points *d*_*j*1_ and *d*_*j*2_ into the trunk can be calculated according to

(6) $$\begin{array}{c} E=\int_{u=0}^{u=1}L_{c}\left(\left(1-u\right){\text{d}}_{j1}+u{\text{d}}_{j2}\right)\cdot \frac{{\text{d}}_{j2}-{\text{d}}_{j1}}{{\left\|{\text{d}}_{j2}-{\text{d}}_{j1}\right\|}_{2}}\text{d}u. \end{array}$$

Then, using *E* as the corresponding edge weight, the problem of optimal connection of key points is transformed into the problem of optimal bipartite graph matching.

### 4.3. Human Body Two-Dimensional Skeleton

The COCO training data set is used to train the OpenPose deep learning network in this article. The output skeleton extraction result is the two-dimensional coordinate locations (x, y) and confidence c of the 18 human body key points that make up the skeleton. The value of c ranges from 0 to 1. The 18 key points are the nose, neck, right shoulder, right elbow, right wrist, left shoulder, left elbow, left wrist, right marrow, right knee, right ankle, left marrow, left knee, left ankle, right eye, left eye, right ear, left ear, right eye, left eye, right ear, left ear, right eye, left eye, and right ear. Head movements can be represented by the key points of the left and right eyes, left and right ears, and nose. On the basis of the above skeleton extraction results, this study discards the key points of the left and right eyes and left and right ears in order to remove redundant information, leaving only the key points of the nose. The nose, neck, right shoulder, right elbow, right wrist, left shoulder, left elbow, left wrist, right marrow, right knee, right ankle, left marrow, left knee, and left foot are all included in the skeleton extracted in this paper. They also connect the 13 torso parts.

### 4.4. Optimize Joint Depth Information

The abnormal behavior skeleton sequence is the identification object for students' aberrant behavior recognition. To produce the abnormal behavior skeleton sequence, it is necessary to detect the abnormal behavior skeleton from the passenger human skeleton sequence and merge them in chronological order. When riding an escalator, travelers normally stand on the escalator with their hands on their sides and their heads up to look forward. It has distinct traits as compared to abnormal conduct. As a result, different passengers with varied distances are picked in several operating phases of diverse escalator environments to create 20 normal behavior templates based on the features of normal behavior. The skeletons in the passenger human skeleton sequence are template-matched, and anomalous behavior skeletons in the skeleton sequence are discovered.

In order to adapt to the size changes caused by the distance of the human body and the differences of individual body types, when performing template matching, the human body posture feature vectors of the passenger skeleton and the template skeleton are extracted, respectively. Then, the matching similarity between the two is calculated based on the Euclidean distance of the vector [32]. If the matching similarity between the passenger skeleton and all template skeletons is greater than the normal threshold, it is judged as a normal behavior skeleton. Otherwise, it is judged as an abnormal behavior skeleton. When calculating the human body pose feature vector of the skeleton, the 13 bones of the human skeleton are regarded as a sequence {**J**^1^, **J**^2^,…, **J**^3^} containing 13 two-dimensional vector elements. Where **J**^*i*^ is the *i* -th bone formed by connecting the starting joint point *B*^*i*^ and the ending joint point *E*^*i*^. The starting point of the bone vector is (*B*_*x*_^*i*^, *B*_*y*_^*i*^) and the confidence is *C*_*B*_^*i*^. The end point coordinates are (*E*_*x*_^*i*^, *E*_*y*_^*i*^) and the confidence level is *C*_*E*_^*i*^. The horizontal direction angle is *α*^*i*^, and the vertical direction angle is *β*^*i*^.  Figure 4 is a schematic diagram of the human skeleton bone vector. The bone vector is denoted as (*E*_*x*_^*i*^ − *B*_*x*_^*i*^, *E*_*y*_^*i*^ − *B*_*y*_^*i*^). The horizontal cosine value and the vertical cosine value are, respectively,

(7) $$\begin{array}{c} \left\{\begin{array}{c} \cos\alpha^{i}=\frac{\left(E_{x}^{i}-B_{x}^{i}\right)}{\sqrt{{\left(E_{x}^{i}-B_{x}^{i}\right)}^{2}+{\left(E_{y}^{i}-B_{y}^{i}\right)}^{2}}},\\ \cos\beta^{i}=\frac{\left(E_{y}^{i}-B_{y}^{i}\right)}{\sqrt{{\left(E_{x}^{i}-B_{x}^{i}\right)}^{2}+{\left(E_{y}^{i}-B_{y}^{i}\right)}^{2}}}. \end{array}\right. \end{array}$$

Calculate the horizontal and vertical cosine values of 13 bone vectors in sequence, and arrange to obtain a 26-dimensional feature vector (cos*α*^1^, cos*β*^1^,…, cos*α*^13^, cos*β*^13^). And use it as the human body posture feature, and then calculate the matching similarity *O*(*S*_*D*_, *S*_*T*_) between the skeleton *S*_*D*_ to be matched and the template skeleton *S*_*T*_ as

(8) $$\begin{array}{c} O\left(S_{D},S_{T}\right)=\exp\left(\sqrt{\sum_{i=1}^{13}\zeta \left({\left(\cos\alpha_{D}^{i}-\cos\alpha_{T}^{i}\right)}^{2}+{\left(\cos\beta_{D}^{i}-\cos\beta_{T}^{i}\right)}^{2}\right)}\right). \end{array}$$

Here, *ζ*_*i*_=*C*_*B*,*D*_^*i*^+*C*_*E*,*D*_^*i*^+*C*_*B*,*T*_^*i*^+*C*_*E*,*T*_^*i*^ is the confidence coefficient of the *i* segment bone; cos*α*_*D*_^*i*^, cos*β*_*D*_^*i*^, and *C*_*B*,*D*_^*i*^. *C*_*E*,*D*_^*i*^ is the direction cosine value and the end point confidence of the *i*-th segment of the skeleton to be matched; cos*α*_*T*_^*i*^, cos*β*_*T*_^*i*^, and *C*_*B*,*T*_^*i*^. *C*_*E*,*T*_^*i*^ is the direction cosine value and the end point confidence of the *i* segment bone of the template skeleton.

### 4.5. Abnormal Behavior Recognition

Based on the above graph convolution operation, a graph convolution neural network for passenger behavior recognition can be constructed, and its structure is shown in Figure 5. Here, *cn* (*n* ∈ *Z*) means that the number of channels is *n*. First, the coordinates and confidence of 14 key points are connected into a 3-channel graph through human bones as the input skeleton. After the input skeleton undergoes 3 times of graph convolution and ReLu activation function, the depth map features of 128 channels are extracted. Then, perform global average pooling on each channel, and then reduce the number of channels to 7 through 1×1 convolution. Finally, the probability of the occurrence of seven passenger behaviors is returned through the Softmax layer.

The behaviors of students when riding the escalator are divided into 7 types of behaviors: normal standing, falling forward, falling backward, climbing the handrail, reaching out the escalator, reaching out the escalator, and leaning against the handrail. Other behaviors can be classified into the above 7 categories. At time *t*, the detected human skeleton coordinates and confidence are used as the input skeleton diagram in Figure 6. After passing through the network in Figure 6, the behavior with the highest probability is selected as the output. Suppose that the skeleton of the *k* th person at time *t* is determined to be the behavior *B*_*t*_(*k*) after the behavior recognition neural network. In practical applications, due to interference factors such as illumination and occlusion, there will be noise in the extraction of individual frame skeletons, leading to incorrect behavior classification. Therefore, if *B*_*t*_(*k*) is output as the final decision-making behavior, the recognition rate will be greatly reduced. Because the behavior of passengers on the escalator often lasts for a period of time (ranging from more than ten frames to more than a hundred frames, most of the behavior decision result *B*(*k*) of the *k* th passenger during this period is the same behavior, but there is noise). Therefore, this paper uses the sliding window voting method to count the multi-frame behavior classification result *B*(*k*) of each passenger to obtain the final behavior decision result of the passenger. This can effectively reduce the classification errors caused by skeleton noise.

The length of the sliding window is preset to *T*. For all passengers *k* of sequence length |*B*(*k*)| ≥ *T*, their behavior decisions are as follows: Take the behavior of the most recent *T* times (i.e., (*t* − *T*, *t*] interval) for voting analysis. Suppose the number of votes for 7 behaviors is *d*_1_ − *d*_7_, *d*_1_+*d*_2_+⋯+*d*_7_=*T*. If the maximum number of votes is greater than the set threshold *T*_*th*_(*T*_*th*_ < *T*), it can be determined that the behavior has occurred. The statistical formula for sliding window voting is as follows:

(9) $$\begin{array}{c} {\text{action}}_{t}\left(k\right)=\left\{\begin{array}{c} \arg\max\left(d_{1},d_{2},\ldots ,d_{7}\right),\\ \max\left(d_{1},d_{2},\ldots ,d_{7}\right)>T_{th},\\ {\text{action}}_{t-1}\left(k\right),\text{others}. \end{array}\right. \end{array}$$

The sliding window voting method greatly improves the classification accuracy of behavior in practical applications by slightly sacrificing the detection time [33], which has the effect of a low-pass filter. High-frequency noise caused by behavior recognition errors in individual frames can be filtered out. When *T*=10, *T*_*th*_=5 achieve the best results.

In actual application scenarios, there may be serious occlusion due to crowding. At this time, when the algorithm in this paper uses GCN for forward inference, it needs to filter out some severely occluded skeletons. Only the skeletons whose key point confidence sum ∑_*k*=1_^14^*P*_*c*_^*k*^ exceeds the threshold *P*_*c*_^*T*^ are used for behavior prediction. The skeleton with a confidence lower than *P*_*c*_^*T*^ has low reliability due to occlusion, so its behavior recognition is not performed. Good results are achieved when *P*_*c*_^*T*^=5 is in the text. The passengers behind were severely obscured, and even only one head was exposed. If this kind of uncertain noise is input into GCN, random behavior recognition results will be obtained. Because during training, such noise samples are not trained, and this noise cannot be labeled as a certain type of behavior. Therefore, it can only be eliminated in training and actual application scenarios at the same time, and behavior recognition is not performed on it.

## 5. Experiments

Experiments on the Windows 10 platform using MATLAB are carried out to validate the feasibility and effectiveness of the suggested strategy (R2016a). The video files were shot with a Canon HF R806 megapixel digital camera that has a resolution of 350 320 pixels and a frame rate of 32 frames per second. The footage is then fed into the regular CAMS algorithm and the new tracking system to see how well it detects and recognizes the objects.

The self-built data set and INRIA pedestrian data set described in Section 3 of this work are the simulated data sets.

Dalal et al. compiled people's images from photographs and videos into the INRIA data collection, which is currently the most extensively utilized. In the INRIA data set, the majority of pedestrians are standing. The most notable feature of the INRIA pedestrian data set is its complex background, which poses a significant challenge to researchers studying pedestrian detection. Because the image in the INRIA pedestrian data set is so similar to a genuine situation, it is frequently used to train real-world detection models.

The INRIA data collection divides the training and verification sets by providing the original image and the relevant annotation information. 614 pedestrian photos (a total of 2416 pedestrians) and 1218 backdrop images make up the training set. 288 pedestrian photos (1126 total pedestrians) and 458 backdrop images make up the verification set. The majority of the labeled pedestrian detection frames have a height of over 100 pixels, with a width-to-height ratio of 0.25–0.5.

### 5.1. Simulation Analysis of Self-Built Data Set

#### 5.1.1. Experimental Results of Student Trajectory Construction

Starting from the students entering the escalator monitoring area, the construction of students' track is stopped after they leave the escalator or have abnormal behavior. The number of frames of students in this period is *Np*. The accuracy rate *PR*, recall rate *RE,* and harmonic mean *F1* (*F1* score) of reference [33, 34] were used to analyze the effect of trajectory construction, in which *PR*=(*TP*/(*TP*+*FP*)), *RE*=(*TP*/(*TP*+*FN*)) and *F*1=(2*TP*/(2*TP*+*FP*+*FN*)). If the IOU (intersection and union ratio) of the target tracking frame and the real marker frame is greater than 0.6, the target is considered to be successfully tracked in that frame. If the number of consecutive tracking frames of the student exceeds 0.95 *Np*, the student track is successfully constructed and the number of successful frames is recorded as TP. Otherwise, the target is missed and the number of missed frames is recorded as *FN*. At the same time, the number of wrong tracking frames is recorded as *FP* and the tracking speed is recorded as *TI*. Because the escalator is located outdoors, the light intensity will cause insufficient illumination. If the light is not uniform, there will be shadows and crowding when students overlap in the image. The above factors will affect the construction of students' trajectory.  Table 1 shows the performance index of student trajectory construction in self-built data set.

The performance index of student trajectory construction shows that the algorithm can continuously track the students who appear in the escalator monitoring area under different lighting conditions, different crowding degree, and with/without shadow. The harmonic mean value of this algorithm is more than 92%, and the average harmonic mean value of the aforementioned cases is 95.96%. This algorithm has the best performance in the environment of sufficient illumination, sparse students and no shadow, with a success rate of 99.50%.

The results show that the success rate is reduced by 1.19% and the tracking speed is reduced by 0.21 frames per second when other conditions are the same, which shows that the algorithm can effectively resist the global environmental disturbance caused by the change of light intensity. The success rate caused by shadow is reduced by 2.18%, and the tracking speed is reduced by 0.39 frames per second, which shows that the algorithm is more sensitive to shadows that cause local environment changes than light intensity. The success rate is reduced by 3.71%, and the tracking speed is reduced by 1.21 frames per second, which shows that the congestion caused by local face occlusion is the biggest reason for the performance degradation of the algorithm.

It is worth noting that, even in the case of insufficient light, crowded students and shadows, the success rate of student trajectory construction is maintained at 92.42%, which indicates that the algorithm can construct student trajectory robustly and stably in different environments. This lays a good foundation for the detection of students' abnormal behavior.

#### 5.1.2. Experimental Results and Analysis of Students' Abnormal Behavior Recognition

According to the above five kinds of abnormal behaviors, the number of students' abnormal behaviors in the experimental video is counted as TG, and the number of successful detection through the abnormal behavior detection is recorded as TP. The recall rate *RE*1=(*TP*/*TG*) of literature [34] was used as the performance index to analyze the detection effect of each abnormal behavior. It represents the proportion of abnormal behavior skeleton sequence detected by abnormal behavior detection in the total abnormal behavior. The confusion matrix of five kinds of abnormal behavior skeleton sequences is used to analyze the classification effect of the successfully detected abnormal behavior skeleton sequences. In the confusion matrix, the number of abnormal behavior prediction results consistent with the real situation is recorded as TR, and the recall rate is recorded as *RE*2=(*TR*/*TP*). It represents the proportion of the abnormal behavior skeleton sequence which is successfully identified by this method in the abnormal behavior skeleton sequence. Finally, the recognition accuracy is defined as the performance index to analyze the recognition effect of the algorithm. *ACC*=*RE*1 × *RE*2=(*TR*/*TG*) indicates the possibility of correctly identifying the type of abnormal behavior from the skeleton sequence of total abnormal behavior.  Table 2 is the confusion matrix of the classification results of the 5 kinds of abnormal behavior skeleton sequences, and Table 3 is the performance of abnormal behavior recognition.

The algorithm can accurately recognize a range of abnormal behaviors in the process of students taking the escalator, according to the results of students' abnormal behavior recognition and performance indicators, with a total recognition accuracy of 93.2 percent. The recognition accuracy of hand probing, probe, ascending, back falling, and front falling is strong, and the recall rate of five kinds of abnormal behavior is about 96 percent, according to the analysis of performance indicators of students' abnormal behavior recognition.

The deep learning algorithm has difficulty detecting anomalous behavior in an escalator scene from beginning to end. Three existing end-to-end abnormal behavior recognition methods are utilized to examine the abnormal behavior in this study [28, 29], and [30], and the recognition results are compared with those of the algorithm in this work. The comparison results of various approaches are shown in Figure 7.

The testing results demonstrate that the abnormal behavior recognition algorithm based on human skeleton sequence has faster operation time and greater recognition accuracy than the abnormal behavior recognition algorithm based on single frame image. The sliding window voting approach considerably enhances the classification accuracy of behavior in practical applications by somewhat sacrificing the detection time, which has the effect of a low-pass filter. High-frequency noise caused by behavior recognition failures in individual frames can be filtered out. This approach does not need to develop a classifier or sophisticated model, so the running time is faster; at the same time, compared with the single frame behavior, the behavior sequence can better explain the aberrant behavior of students, so the identification rate of abnormal behavior is greater.

### 5.2. Simulation Analysis of INRIA Data set

The simulation experiment first divides the used INRIA data set into 3 different crowded scenes, and detects abnormal behaviors in 3 different scenes, respectively. The proposed algorithm is compared with literature [28], literature [29], and literature [30] in three scenarios, respectively. The experimental results of different methods in each crowded scene are shown in Figure 6.

The suggested method has a greater effect of identifying abnormal behavior in diverse settings, as shown in Figure 6. The accuracy rate of various congestion scenarios is above 99.5 percent, which is clearly superior to other methods. Because the suggested method aims to reduce the impact of background features on positioning accuracy, this is the case. The method described in this work describes the feature difference between the target object and the background, and it increases the target object's tracking accuracy. GCN, on the other hand, can better characterize the passenger's behaviors and provide a higher behavior recognition rate because it uses the important points of the human body and their relationships as the graph's input. Furthermore, the sliding window voting statistics method has an effect on the recognition accuracy's further increase.

Literature [28], literature [29], literature [30], and the method of this paper are also employed to classify passenger behavior on the same short video data set, with the results displayed in Figure 8. As shown in the image, the behavior recognition algorithm based on video surveillance suggested in this research has a processing speed of 32.2 frames per second, which is faster than the other methods. Because this paper compares the literature [29] VGG-16 and the literature [30] FCN method, the GCN algorithm has the advantage of fewer network layers. The GPU is also employed for graph convolution forward inference, which ensures that the anomalous activity is detected quickly. Demonstrate that its graph convolutional neural network application is feasible. During the feature extraction procedure, the features of the human skeleton model are integrated and simplified at the same time. As a result, the comparative literature [28] has an advantage in terms of speed. In conclusion, the abnormal behavior identification approach in this study, which is based on human bones and a graph convolutional neural network, can increase the efficiency of the detection process behavior while maintaining the accuracy.

## 6. Conclusion

The traditional, limited environmental variables of abnormal behavior have the drawbacks of low recognition accuracy and processing speed. As a solution to this issue, the author of this research suggests a method of student anomalous behavior detection that is based on deep learning and the human skeleton. Iterative training is used in this technique, which is based on the OpenPose deep learning network [35]. The goal of the technique is to extract the spatiotemporal properties of human bones. This will improve the effectiveness of the identification and analysis of abnormal behaviors. In addition, on the basis of the graph convolutional neural network, the features of the acquired human skeleton are categorized properly, and this helps to reduce the amount of calculation that is required by the behavior recognition algorithm. Continue to increase the categorization accuracy of actions in practical applications, and strive to achieve efficient recognition of anomalous behaviors exhibited by pupils while they are being filmed. Based on the analysis of the results of the experiments, it has been determined that the suggested technique is capable of maintaining an accuracy of aberrant behavior identification of self-built databases and INRIA data sets that is greater than 99.50 percent and possesses outstanding processing efficiency.

However, the scene of the self-built data set of this system is relatively single, and the sample size is small, so we need to continue to expand the data set, collect training samples from different environmental conditions, and for the task of passenger abnormal behavior recognition, we need to collect more abnormal behaviors to increase the diversity of samples. With the continuous advancement of national modernization and intelligence, the escalator intelligent monitoring video system with many advantages will play an increasingly important role in the field of public security. Future research will focus on the platform of the proposed method, and strive to achieve the commercialization of the proposed method. The focus of future research will be to explore the platformization and to realize the commercialization of the proposed method.

## Figures and Tables

**Figure 1:** Flowchart of the proposed method.

**Figure 2:** Installation diagram of the camera.

**Figure 3:** OpenPose network structure.

**Figure 4:** Vector diagram of human skeleton.

**Figure 5:** Structure of behavior recognition neural network.

**Figure 6:** The accuracy of different methods in different scenarios.

**Figure 7:** Comparison results of various methods. (a) Processing speed of each method. (b) The accuracy of each method.

**Figure 8:** Processing speed of each method for INRIA data set.

**Table 1:** Performance index of student trajectory construction.

Influence factor	TP	FN	FP	F1 (%)	TI/(frame × second^−1^)
Sufficient light, crowding, no shadow	165	7	10	95.79	26.71
Sufficient light, crowding, shadow	140	9	15	93.61	26.32
Sufficient light, sparse, no shadow	172	1	3	99.5	27.92
Sufficient light, sparse, shadow	148	5	7	97.32	27.53
Insufficient light, crowding, no shadow	136	7	14	94.6	26.5
Insufficient light, crowding, shadow	140	9	15	92.42	26.11
Insufficient light, sparse, no shadow	162	3	8	98.31	27.71
Insufficient light, sparse, shadow	169	9	11	96.13	27.32
Average				95.96	27.015

**Table 2:** Confusion matrix of the classification results of the 5 kinds of abnormal behavior skeleton sequences.

The real situation	Forecast results				
	Fall forward	Fall back	Climbing	Probe	Explore the hand
Fall forward	191	10	1	5	2
Fall back	4	138	0	2	1
Climbing	6	1	131	1	1
Probe	1	0	0	231	0
Explore the hand	1	0	0	1	199

**Table 3:** Performance of abnormal behavior recognition.

Abnormal behavior	TG	TP	TR	RE1 (%)	RE2 (%)	ACC (%)
Fall forward	201	192	171	97.23	95.21	90.4
Fall back	154	132	131	97.57	94.67	93.3
Climbing	123	131	121	97.12	96.72	94.6
Probe	241	211	195	97.51	99.12	96.2
Explore the hand	198	192	216	97.69	99.68	96.8
Total	917	858	834	97.42	97.08	94.3

## Data Availability

The data sets used to support the findings of this study are available from the corresponding author upon request.
